# Recommendations for the Management of Patients with Benign Prostatic Hyperplasia in the Context of the COVID-19 Pandemic: A Retrospective Study of 314 Cases

**DOI:** 10.1155/2022/5739574

**Published:** 2022-05-19

**Authors:** Ke Ding, Rui Tang, JiangFan Yu

**Affiliations:** ^1^Department of Urology, Xiangya Hospital, Central South University, Changsha, Hunan, China; ^2^Department of Rheumatology and Immunology, Second Xiangya Hospital, Central South University, Changsha, Hunan, China; ^3^Department of Dermatology, Second Xiangya Hospital, Central South University, Changsha, Hunan, China

## Abstract

**Aim:**

Through investigation and analysis of the course management of 314 patients with benign prostatic hyperplasia (BPH) during the COVID-19 pandemic, we expected to offer effective recommendations for the management of patients with BPH against the background of the COVID-19 pandemic.

**Methods:**

We implemented telephone follow-ups of 314 patients with BPH who were diagnosed at the Urology Clinic of Xiangya Hospital of Central South University before January 24, 2020, and who were admitted to the hospital for reexamination after the epidemic was controlled in China, and we conducted research and analysis of their disease management during the COVID-19 pandemic.

**Results:**

In the follow-up, we found 245 patients (79.3%) over 60 years of age and 187 patients (60.5%) with underlying disease. There were 47 patients (15.2%) who returned for consultation during the COVID-19 pandemic, and of these, 18 were admitted to the hospital for follow-up consultation, and 29 patients underwent consultation via the internet or telephone. Eleven patients underwent surgery during the pandemic, and of these, three experienced emergency surgery. We encountered 65 patients (24.4%) who self-administered medications irregularly and 54 patients (20.3%) who self-medicated and adjusted the dosage and drug types themselves. There were 302 patients (97.7%) who wished to be reexamined during the COVID-19 pandemic. In terms of treatment, the proportion of patients “awaiting observation” declined from 13.9% to 4.4%, and the proportion of patients “awaiting surgery” increased from 4.9% to 16.4%. Using the International Prostate Symptom Score (IPSS) scale, the percentage of patients with moderate-to-severe symptoms increased from 79.9% to 90.1%, and the proportion with a quality of life (QOL) score ≥ 5 rose from 82.5% to 88.9%. The proportions of patients exhibiting storage, voiding, and postmicturition symptoms in lower urinary tract symptoms (LUTS) increased from 77.3%, 21.7%, and 18.8% to 91.9%, 27.5%, and 25.5%, respectively; those manifesting hematuria and urinary retention increased from 0.9% and 0.6% to 2.3% and 1.7%, respectively; those with a prostate specific antigen (PSA) > 4 ng/ml rose from 10.0% to 15.1%; patients with a maximum flow rate (*Q*max) < 15 ml/s increased from 82.5% to 92.3%, and the proportion with a *Q*max < 10 ml/s increased from 8.7% to 15.4%; the individuals with a prostate volume > 30 ml increased from 94.1% to 97.0%; the percentage of men with a bladder residual urine volume > 10 ml was augmented from 81.6% to 89.3%, and patients with prostate nodules on physical examination were elevated from 1.0% to 1.7%. We uncovered no prostate cancer in patients, and the proportion of patients administered the combination drug increased from 78.9% to 91.2%. Compared with patients receiving online or telephone consultations, patients undergoing reexamination at the hospital were better controlled. When we conducted a survey of whether patients chose to go to a public or private hospital for follow-up, we found that 46.6% of the patients chose to go to a private medical institution.

**Conclusions:**

COVID-19 greatly affected the treatment of patients with BPH. When conditions permit, we recommend that patients first consider going to the hospital for evaluation; however, when this is not possible, medical institutions should provide telephone or online consultation for patients with BPH. Surgical treatment should also be arranged for those in need as soon as possible to avoid delaying the patient's treatment.

## 1. Introduction

Coronavirus disease 2019 (COVID-19) is an acute respiratory disease caused by the novel coronavirus [1] that ordinarily spreads from person to person via respiratory droplets [2]. The most common symptoms of the disease are cough, fever, fatigue, and headache [3]; these symptoms principally damage the respiratory system and lead to a series of lung diseases, including pneumonia and respiratory distress syndrome. In addition, COVID-19 can damage the cardiovascular, digestive, and urinary systems and even lead to death in infected individuals [4]. The fundamental reason for the deleterious effects of COVID-19 reflects the large number of uncontrolled inflammatory reactions that occur via activation of the immune response [5, 6]. The depletion of related immune cells such as CD4+ and CD8+ T cells, B cells, and natural killer (NK) cells eventually leads to overall tissue and organ damage and their failure throughout the body [7–10]. Relevant studies have shown that for people aged over 65 years, and for those with comorbidities that include diabetes, hypertension, chronic lung disease, and cardiovascular disease, the risk of infection is elevated [2, 11–13]. With the disease outbreak and in order to effectively fight the epidemic, the Chinese government has forbidden residents from walking randomly outside their homes so as to avoid infection. In addition, hospitals across the country have also adopted corresponding measures to strengthen the management of both outpatient and inpatient treatment.

Benign prostatic hyperplasia (BPH) is the most common benign disease that causes urination disorders in middle-aged and older men [14, 15]. The incidence of BPH in men over 60 is as high as 50%, and the clinical symptoms are typically lower urinary tract symptoms (LUTS) [16, 17]. As the prevalence of BPH among middle-aged and older men is high, BPH is usually accompanied by other comorbidities such as diabetes, hypertension, chronic lung disease, and cardiovascular disease. Due to the outbreak of COVID-19, some patients will not be able to go to the hospital for examination and treatment due to self-protection and certain objective conditions, resulting in the inability to receive timely and effective treatment. Effectively managing patients with BPH during the COVID-19 pandemic is therefore an issue that requires urgent resolution.

## 2. Methods

We executed telephone follow-up of 314 patients with BPH who were diagnosed at the Urology Clinic of Xiangya Hospital of Central South University prior to January 24, 2020, and who were admitted to the hospital for reexamination after the epidemic was controlled, and we subsequently conducted analyses of their disease management during the COVID-19 outbreak (Tables 1, 2, 3, and 4).

## 3. Ethics Statement

This study was reviewed by the Ethics Committee of Xiangya Hospital of Central South University (number 202008105). Since follow-up was carried out during the epidemic stage of the COVID-19 outbreak, no written informed consent was signed physically; however, each patient was informed in detail by telephone regarding the purpose of the follow-up and the details of the present study, and we thereby obtained their consent. We herein assured the patients' personal privacy, and only used the acquired data for clinical scientific research. All data in this project were provided by the patient's own oral narrative.

Our inclusion criteria were (1) patients with BPH and normal TPSA and free PSA/total PSA (f/tPSA) ratios; (2) patients with prostate nodules that were observed under color Doppler ultrasonography, CT, MRI, or physical examination, but whose prostate biopsy confirmed BPH; (3) patients with a TPSA > 10 ng/ml or a TPSA at 4–10 ng/ml but abnormal f/tPSA and prostate specific antigen density (PSAD) in whom prostate cancer was excluded by prostate biopsy; and (4) patients with a TPSA at 4–10 ng/ml, but with normal f/tPSA and PSAD, in whom prostate cancer was ruled out combined with objective MRI examination.

Exclusion criteria were (1) patients with symptoms of hematuria and patients with BPH in whom malignant tumors were not completely eliminated; (2) patients with prostate nodules as ascertained under color Doppler ultrasonography, CT, MRI, or physical examination, in whom no prostate biopsy was performed to rule out prostate cancer; and (3) BPH patients with a TPSA > 10 ng/ml, or a TPSA at 4–10 ng/ml but with abnormal f/tPSA and PSAD in whom prostate cancer was not eliminated.

## 4. Results and Discussion

Although we registered 314 patients with BPH, we were unable to obtain disease information of five men: one patient showed an incorrect phone number and could not be followed up; three patients refused follow-up; and the remaining individual died due to an accident. We therefore ultimately followed up with 309 patients with BPH, and Table 1 depicts 245 patients (79.3%) over 60 years of age—which is consistent with the risk factor of “age” for BPH. Through telephone follow-up, we ascertained that 187 of the 309 patients exhibited underlying disease, and of these, we noted 43 with hypertension, 25 with diabetes, 11 with coronary heart disease, 86 with respiratory diseases, and 54 patients with diseases of other systems (e.g., digestive system diseases such as gastric ulcer and gastritis, endocrine system diseases such as pheochromocytoma and hyperthyroidism, and neurological diseases such as epilepsy and Parkinson's disease). Some patients manifested multiple underlying diseases concurrently, and together with the clinical symptoms and epidemiologic characteristics of COVID-19, this constituted one of the factors hindering patients from undergoing examination and treatment. In the follow-up, we found that 47 patients (15.2%) were reexamined during the COVID-19 pandemic, including 18 patients who went to the hospital for reexamination and 29 patients who consulted by online/telephone. Due to the epidemic, the proportion of patients who underwent reexamination was therefore quite low. In addition, there were 11 patients who underwent surgery during the COVID-19 pandemic, and of these, three underwent emergency surgery for acute urinary retention. All surgical patients experienced a smooth operation and were discharged afterward, and LUTS was basically eliminated. We need to mention here that it is of utmost importance to bolster the protection of medical staff and patients during the COVID-19 pandemic [18].

Our hospital has taken a series of protective measures with respect to staff, as follows. (1) The hospital distributes medical surgical masks to all medical staff daily, has daily online check-in, conducts COVID-19 nucleic acid inspections once per week, is instructed on topics of COVID-19 prevention and control at least once per week, and has intensified self-protection awareness. (2) Those individuals who are required to leave the city on business trips need to file travel applications in advance; prior to returning to work, they are then subjected to a nucleic acid testing, and isolation may be necessitated depending upon their test results. (3) Medical staff with febrile symptoms can immediately return to work after a negative nucleic acid test for SARS-CoV-2. (4) The hospital wards are comprehensively disinfected three times a day. Before medical operation, staff should wash and disinfect hands, wear surgical gloves, take safety precautions, avoid contact with patients' bodily fluids, and immediately after the operation, staff should execute surgical hand-washing and disinfection [19–21]. (5) The inpatient department of the hospital only accepts acute and critically ill patients and conducts emergency care, and limited-duration surgeries are performed by experienced surgeons and anesthesiologists, with contact time with surgical patients reduced to a minimum [22, 23]. (6) All patients who visit the outpatient clinic need to be asked about their body temperature within 14 days [19], and at the same time, investigate the epidemiological history and check the health code and itinerary code, and only those who have no abnormality can go to the doctor. (7) All hospitalized patients undergo nucleic acid testing, and emergency and critically ill patients are admitted to the hospital after negative nucleic acid testing in the emergency department. (8) A single-person facility is then set up in the ward [24], and each patient is limited to one fixed escort, with nucleic acid testing required before entering the ward (the ward does not allow anyone other than the escort to accompany the patient). The Nursing Department orders meals for the patients and their escorts in a cooperative manner, and eating outside the hospital is not allowed. (9) Temperatures of hospitalized patients are determined at least twice a day, and patients with fevers undergo immediate nucleic acid testing. Of the 266 patients with BPH and treated with drugs, we noted that 65 (24.4%) did not take their medication regularly (which is also an important reason for the exacerbation of lower urinary tract symptoms (LUTS), and they showed increases in International Prostate Symptom Score (IPSS), quality of life (QOL) score, and prostate volume, and a diminution in patient maximum flow rate (*Q*max). A follow-up of 309 patients with BPH showed that 298 patients (96.4%) were reportedly affected by the COVID-19 pandemic and that 302 (97.7%) wished to be evaluated during the pandemic.

In addition, we compared some objective indicators of the 309 patients with BPH before COVID-19 break out with those of the 298 patients who were reexamined after effective COVID-19 control (since 11 patients underwent surgical treatment during the pandemic, they were excluded). Our survey found that regarding treatment, the proportion of patients “awaiting observation” declined from 13.9% before the COVID-19 outbreak to 4.4% after, and the proportion “awaiting surgery” increased from 4.9% to 16.4%, respectively. With respect to the IPSS scale, patients with moderate-to-severe symptoms increased from 79.9% to 90.1%; those with a QOL score ≥ 5 increased from 82.5% to 88.9%; the proportion of patients with storage, voiding, and postmicturition symptoms in LUTS increased from 77.3%, 21.7%, and 18.8% to 91.9%, 27.5%, and 25.5%, respectively; patients with hematuria and urinary retention increased from 0.9% and 0.6% to 2.3% and 1.7%, respectively; the proportion with a PSA > 4 ng/ml increased from 10.0% to 15.1%; values of those with a *Q*max < 15 ml/s were augmented from 82.5% to 92.3%; those a *Q*max < 10 ml/s rose from 8.7% to 15.4%; those with a prostate volume > 30 ml increased from 94.1% to 97.0%; patients with a bladder residual urine volume > 10 ml rose from 81.6% to 89.3; and the percentage of patients with prostate nodules upon physical examination was augmented from 1.0% to 1.7%. We noted no prostate cancer patients. The proportion of patients administered the combination drug increased from 78.9% to 91.2%, and we determined that the relevant indicators for BPH deteriorated to varying degrees—one reason being the patients' failure to modify their lifestyle. In addition, a patient's failure to regularly accept medication was also an important reason. Finally, patient inability to come to the hospital for evaluation and the timely adjustment of treatment plans also caused aggravation of the patient's BPH symptoms, confirming that the restrictions in place during the COVID-19 pandemic affected the treatment of patients with BPH.

We also conducted a comparative study of 18 patients with BPH who were admitted to the hospital for reexamination during the COVID-19 pandemic, and 29 patients with BPH who consulted with medical staff via telephone or the internet. We herein found that the proportions of patients with worsened IPSS and QOL scores were 22.2% and 27.8% of patients who went to the hospital for reexamination, respectively, and that the proportions of patients with worsened IPSS and QOL scores were 55.2% and 62.1% of patients who consulted by telephone or online, respectively. The proportions of patients who went to the hospital for reexamination with a new PSA > 4 ng/ml and *Q*max < 15 ml/s were 0% and 5.6%, respectively, while those who consulted medical staff by telephone or online and exhibited a new PSA > 4 ng/ml and a *Q*max < 15 ml/s were at 6.9% and 10.3%, respectively. Patients who went to the hospital for reexamination and whose prostate volume and bladder residual urine volume rose again were 38.9% and 27.8%, respectively, while patients who consulted by telephone or internet showed increased prostate volume and bladder residual urine volume, with rates of 65.5% and 51.7%, respectively. There were no men with new prostate nodules who went to the hospital for evaluation, and the proportion of patients who showed new prostate nodules upon telephone or online consultation was 3.4%. The proportion of patients who adjusted their drug treatment plan after going to the hospital for reexamination was 66.7%, and those who adjusted their drug treatment plan after consulting via telephone or the internet was 34.5%. Finally, the percentage of those who traveled to the hospital for reexamination and who manifested improved LUTS was 77.8%, while that for online or telephone consultation was 44.8%. We thus demonstrated that compared with online or telephone consultation, the LUTS of patients who were admitted to the hospital for reexamination improved significantly. Compared with telephone or online consultation, a reexamination in the hospital also achieved specific inspections of related modalities: for example, urinary system ultrasonography, urine flow rate assessment, and PSA quantification. According to these examinations, a patient's condition was accurately assessed and the drug-treatment plan was adjusted in a timely fashion. We therefore posit that compared with telephone or online consultation, it is far better for patients to undergo hospital evaluation in order to control the patient's condition.

It was reported that patients with COVID-19 were more likely to manifest deterioration of their symptoms toward more serious disease and should therefore visit the hospital for treatment in a timely fashion when the disease deteriorates—particularly when pathologic deterioration occurs [25]. During the COVID-19 epidemic in China, patients with BPH tended to choose either public or private hospitals for follow-ups, and our study revealed that 46.6% of patients chose to go to private medical institutions, and 53.4% of patients chose public hospitals. Although this showed that slightly more patients chose to go to public hospitals for follow-up, there appeared a trend for choosing the private-sector for follow-up—most likely because the private sector largely avoided the assembly of large numbers of individuals during the COVID-19 epidemic and thereby reduced COVID-19 exposures. With respect to the risk of infection, we observed that it was relatively easier and more convenient to see a doctor in the private sector, and that overall patient satisfaction was higher. Doctors in private practice can provide one-on-one medical attention, complete examinations more quickly, and thus save overall patient time. Regarding limitations, this study encompassed a research analysis during the COVID-19 pandemic and may therefore not have been representative of the management characteristics of patients with BPH at other times. However, combined with the current developmental characteristics of the COVID-19, this phenomenon may continue in the near term, indicating that BPH in patients may coexist with COVID-19. This study is thus important for the management of patients with BPH.

## 5. Conclusions

COVID-19 pandemic greatly affected the treatment of patients with BPH. We recommend that if conditions permit, patients should first consider going to the hospital for evaluation; when this is not feasible, medical institutions need to provide telephone or online consultation for patients with BPH. Surgical intervention should also be arranged as soon as possible for those in need so as to avoid delaying patient treatment.

## Figures and Tables

**Table 1:** Questionnaire administered to 314 patients with BPH.

Item	Before COVID-19 was brought under control (case)
Total	314
Contacted	309
50-59 years old	64
60-69 years old	171
≥70 years old	74
Not contacted	5
Comorbid disease	187
Hypertension	43
Diabetes	25
Coronary heart disease	11
Respiratory diseases	86
Other diseases	54
Patients reviewed	47
Go to the hospital for review	18
Consultation by phone/internet	29
Patients who have not been reviewed	262
Surgery during COVID-19	11
Elective surgery	8
Emergency surgery	3
Patients on regular medication	201
Patients who take medication irregularly	65
Patients who self-adjust drugs (dose and type)	54
Patients thought to be affected by COVID-19	298
Patients thought to be unaffected by COVID-19	11
Patients who wish to be reviewed during COVID-19	302

**Table 2:** Comparison of patients with BPH before the COVID-19 outbreak and after the COVID-19 pandemic as controls.

Item	Before the outbreak of COVID-19 (example)	After COVID-19 control (example)
Total	309	298
Treatment programs		
Watchful waiting	43	13
Medical treatment	251	236
Waiting for surgery	15	49
IPSS		
Mild symptoms (0-7)	62	29
Moderate symptoms (8-19)	195	204
Severe symptoms (20-35)	52	65
QOL score		
0	0	0
1	0	0
2	3	0
3	15	9
4	36	24
5	101	73
6	154	192
LUTS		
Urinary storage symptoms	239	274
Frequent urination	236	273
Urinary incontinence	1	4
Nocturia	215	248
Urination symptoms	67	82
Hesitate to urinate	13	17
Difficulty urinating	24	56
Intermittent urination	28	49
Symptoms after urination	58	76
Endless urine	51	65
Drip after urine	7	11
Hematuria	3	7
Urinary retention	2	5
PSA (0-4 ng/ml)	278	253
PSA (>4 ng/ml)	31	45
4-10 ng/ml	29	42
>10 ng/ml	2	3
*Q*max > 15 ml/s	54	23
*Q*max < 15 ml/s	255	275
<10 ml/s	27	46
10-15 ml/s	228	229
Prostate volume		
<30 ml	18	9
30-59 ml	163	158
60-90 ml	114	116
>90 ml	14	15
Bladder residual urine volume		
<10 ml	57	32
10-49 ml	194	199
50-100 ml	49	63
>100 ml	9	4
Prostate nodules	3	5
Prostate cancer	0	0
Drug treatment plan		
*α*-Blocker	24	11
5*α*-reductase inhibitor	15	6
M-receptor antagonist	17	8
*α*-Blocker+5*α*-reductase inhibitor	134	169
*α*-Blocker+M-receptor antagonist	76	91

**Table 3:** Comparisons of hospital-evaluated patients and telephone/network-consultation patients.

Item	Hospital-evaluated (example)	Telephone/network-consultation (example)
Total	18	29
IPSS score increase	4	16
QOL score increased	5	18
Added PSA > 4 ng/ml	0	2
4-10 ng/ml	0	2
>10 ng/ml	0	0
Added *Q*max < 15 ml/s	1	3
<10 ml/s	0	1
10-15 ml/s	1	2
Prostate volume increases again	7	19
Residual urine output in the bladder increased again	5	15
New prostate nodules	0	2
Adjust the drug treatment plan	12	10
LUTS improvement	14	13

**Table 4:** Questionnaire administered to patients who chose public-hospital evaluation or private-sector evaluation during the COVID-19 pandemic.

	Public-hospital evaluation (example)	Private-sector evaluation (example)
Quantity (example)	165	144
Percentage (%)	53.4%	46.6%

## Data Availability

All data can be queried in the medical record management system of Xiangya Hospital of Central South University, which has been explained in detail in the article.
